# PLCE1 promotes myocardial ischemia–reperfusion injury in H/R H9c2 cells and I/R rats by promoting inflammation

**DOI:** 10.1042/BSR20181613

**Published:** 2019-07-05

**Authors:** WenHua Li, Yong Li, Ying Chu, WeiMin Wu, QiuHua Yu, XiaoBo Zhu, Qiang Wang

**Affiliations:** 1 Department of Cardiology, Wujin People’s Hospital of Changzhou, Changzhou 213017, China; 2 Central Laboratory, Wujin People’s Hospital of Changzhou, Changzhou 213017, China; 3 Department of Cardio-Thoracic, Wujin People’s Hospital of Changzhou, Changzhou 213017, China

**Keywords:** Inflammation, Myocardial ischemia-reperfusion injury, NF-κB, PLCE1

## Abstract

Myocardial ischemia–reperfusion (I/R) injury is a major contributor to the morbidity and mortality associated with coronary artery disease. How to ensure the recovery of blood supply to ischemic myocardial tissue while avoiding or reducing I/R injury remains a critical problem in clinical practice. In the present study, we examined the function of phospholipase C ϵ-1 (PLCE1) by an H9c2 H/R (H/R, hypoxia–reoxygenation) model and a rat myocardial I/R injury model. The expression of PLCE1 and its effect on I/R injury-induced inflammatory response as well as its possible underlying mechanism were investigated. Our results have shown that PLCE1 was progressively increased along with the increase in hypoxia time in the H/R H9c2 and HL-1 cells. In myocardial I/R rats, PLCE1 presented a low expression level in the sham group, however, it was increased sharply in the I/R group. Overexpression of PLCE1 promoted the expression of IL-6, TNF-α, and IL-1α, and decreased the expression of IL-10. Knockdown of PLCE1 decreased the expression of IL-6, TNF-α, and IL-1α, and increased the expression of IL-10. Furthermore, overexpression of PLCE1 increased the phosphorylation of p38, ERK1/2, and nuclear factor-κ B (NF-κB) P65 while knockdown of PLCE1 inhibited their phosphorylation. In conclusion, the present study provided evidence that PLCE1 was up-regulated in H/R H9c2 cell and I/R rat. Overexpression of PLCE1 promoted the inflammatoion via activation of the NF-κB signaling pathway.

## Introduction

In recent decades, cardiovascular diseases such as acute myocardial infarction (AMI) have become the leading cause of deaths in the world [1]. The current clinical management of patients with AMI mainly focused on antiplatelet, thrombolysis (urokinase, streptokinase etc.), and direct percutaneous transluminal coronary angioplasty (PTCA) to reduce the infarct range and rescue the dying cardiomyocytes for hypoxia and insufficient energy supply [2,3]. It is often accompanied by myocardial ischemia/reperfusion (I/R) injury during the treatment and natural turnover course of AMI, which results in a large range of cardiomyocytes death. The process of reperfusion accelerates the death of the severely injured cells and induces a strong inflammatory response which is characteristic of inflammatory cell infiltration and inflammatory cytokine production, eventually leading to myocardial infarction, fibrosis, cardiac hypertrophy, and heart failure [4–6]. Therefore, besides the degree of recanalization of blood vessels, I/R injury has become another important factor affecting the therapeutic effect of AMI.

Recent studies found that the level of inflammatory cytokines is related to the damage of cardiac function and necrosis of cells post ischemia. The inflammatory response plays an important role in myocardial I/R injury, and it has been proved that the I/R-induced injury improved when inflammation was inhibited by the anti-inflammatory agents [7–9]. Nuclear factor-κ B (NF-κB) is a nuclear protein factor, originally found in B lymphocyte nuclear extracts, that binds to the immunoglobulin κ-chain gene enhancer κB sequence and generally presents in the cytoplasm in the form of a heterodimer (P50 and P65) [10]. When suffering from inflammatory stimulation, the NF-κB is activated by phosphorylation of the IκB kinase (IKK) and translocated from the cytoplasm into the nucleus, and then bound to DNA, resulting in inducing the expression of a variety of inflammatory genes [11,12]. Studies have shown that the NF-κB pathway is involved in the pathophysiological process of I/R injury [13,14].

Phospholipase C ϵ-1 (PLCE1) was discovered as a new member of the phosphoinositide-specific PLC family which can be activated by a variety of intracellular and extracellular signal molecules [15]. PLCE1 catalyzes the hydrolysis of phosphatidylinositol-4,5-bisphosphate (PIP2) on the cell membrane to produce two-second messengers, inositol-1,4,5-triphosphate (IP3) and diacylglycerol (DAG). IP3 induces the release of Ca^2+^ in cells and DAG can activate protein kinase C (PKC), which causes phosphorylation of serine and threonine residues on various target proteins in the cytoplasm, thereby regulating cell growth, differentiation, and gene expression [16–18]. Recently, the involvement of PLCE1 in various cancers has become an area of intense interest. Numerous studies have suggested that PLCE1 plays a key role in the development and progression of cancer through various pathways. Therefore, PLCE1 is considered to be a potential target for cancer prevention and treatment [19]. In addition, studies have shown that PLCE1 is also involved in the progression of inflammation and stimulate the expression of a variety of inflammatory cytokines, such as TNF-α, IL-4, IFN-γ etc. [20]. However, the relationship between PLCE1 and myocardial I/R injury has not been reported yet. In the present study, we first explore the biologic functions of PLCE1 and its underlying mechanism in myocardial I/R injury by an H9c2 hypoxia–reoxygenation (H/R) model and a rat I/R model.

## Methods

### Cell lines and animals

The rat heart-derived cardiac myoblast H9c2 cell and mouse heart-derived HL-1 cell were obtained from ATCC (MD, U.S.A.). These cells were propagated in DMEM added with 10% FBS and 1% antibiotics (penicillin 100 U/ml and streptomycin 100 mg/ml) at 5% CO_2_ and 37°C.

Male Sprague–Dawley rats (200 ± 10 g, 8 weeks) were obtained from the Model Animal Research Center of Wujin People’s Hospital of Changzhou (Changzhou, China). The rats were housed in a standard laboratory condition (temperature 22 ± 2°C; humidity 40–60%; 12/12-h light/dark). Rats were fed with the standard chow diet and water *ad libitum*. All animal experiments were performed in accordance with the guidelines of the Experimental Research Institute of Wujin People’s Hospital of Changzhou. This animal experiment was approved by the Medical Ethics Committee of Wujin People’s Hospital of Changzhou.

### *In vitro* H/R model

A controlled hypoxia plastic chamber was used to control the hypoxia time. Briefly, the seeded H9c2 cells were placed in an anaerobic chamber with the anoxic atmosphere at 2.5% O_2_, 5% CO_2_, and 92.5% N_2_ and incubated for 2–24 h at 37°C. Then the cells were reoxygenated under normoxic conditions (95% air/5% CO_2_) for 24 h at 37°C. The control group cells without hypoxia treatment were kept in normoxic conditions.

### Cell viability

Cell Counting Kit-8 (CCK-8) assay was used to evaluate the cell viability of H9c2. Briefly, the cell suspensions were planted in a 96-well culture plate at 4 × 10^3^ cells/well. Overnight, the cells conducted H/R treatment for 2–24 h according to the method described above. After that, 10 μl CCK-8 solutions were added and incubated at 37°C for additional 2–4 h. Then, the absorbance was recorded at 450 nm by a microplate reader (Bio-Rad).

### PLCE1 overexpression vector construction

The cDNA for PLCE1 gene was synthesized and cloned, then it was cloned into a commercial pcDNA3.1 vector (Invitrogen, CA, U.S.A.) as per the manufacturer’s instructions. The cDNAs were then cloned into a lentivirus vector pBabe-puro at Sal I and BamH I sites (pBabe-puro-PLCE1). The PLCE1 expression and control vector were prepared by transient transfection in 293T cells.

### PLCE1 shRNA construction

For knockdown of PLCE1, the shRNA against PLCE1 was designed and synthesized by GenePharma (Shanghai, China). Then the shRNA was cloned into a lentivirus vector pLKO.1 at Age I and Ecor I sites (pLKO.1-PLCE1). A control shRNA without any specific target was used as a negative control (pLKO.1).

### Transfection

Before the H9c2 cells conducted H/R treatment, the PLCE1 expression or knockdown vectors were transfected. Briefly, the cell suspensions were planted in a six-well culture plate at 2 × 10^5^ cells/well. When the cells were covered at 60–80% of the bottom surface of the culture plates, the vectors of pBabe-puro, pBabe-puro-PLCE1, pLKO.1, and pLKO.1-PLCE1 were transfected into the cells by Lipofectamine™ 2000 kit according to the manufacturer’s instructions. After successful transfection, the H/R treatment was continued according to the method described above.

### Western blot

The Western blot assay was conducted as described previously [21]. In brief, the cells or tissues were lysed with RIPA lysis buffer containing 1 mmol/l PMSF. Then the homogenates were prepared and centrifuged at 12000 rpm for 10 min at 4°C. The protein concentration was determined by BCA method. Nonspecific binding was blocked with 5% skimmed milk for 1.5 h, and the membranes were incubated with diluted primary antibodies (PLCE1, NF-κB P65, p-NF-κB P65, P38, p-P38, ERK1/2, p-ERK1/2, and β-actin) overnight at 4°C and in the secondary antibody for 1 h at room temperature. The signals were determined by Amersham prime ECL Plus detection system (Pittsburgh, PA).

### RNA isolation and quantitative polymerase chain reaction analysis

The total RNAs of the cells or tissues were extracted by RNA extraction kit according to the instructions. The reverse transcription was performed with a SuperScript III First-Strand Synthesis system. Quantitative assay of gene expression was performed by a SYBR qPCR Kit (Osaka, Japan). The gene expressions were normalized to the GAPDH and calculated by the Δ*C*_T_ method. The specific primer sequences were listed in Table 1.

**Table 1:** The primer sequences of genes

Genes	Primer sequences
*PLCE1*	F: 5′-GAGCTGCAATCGAAGTCTGG-3′
	R: 5′-GAGCTGCAATCGAAGTCTGG-3′
*IL-6*	F: 5′-TAGTCCTTCCTACCCCAATTTCC-3′
	R: 5′-TAGTCCTTCCTACCCCAATTTCC-3′
TNF-α	F: 5′-GGCTTTCCGAATTCACTGGAG-3′
	R: 5′-CCCCGGCCTTCCAAATAAA-3′
*IL-1α*	F: 5′-GCATCCTCACAGCAGGATTT-3′
	R: 5′-GAATCCAGGGGAAACACTGA-3′
*IL-10*	F: 5′-ATGCCCCAAGCTGAGAACCAAGACCCA-3′
	R: 5′-TCTCAAGGGGCTGGGTCAGCTATCCCA-3′
*GAPDH*	F: 5′-GGGAAATTCAACGGCACAGT-3′
	R: 5′-AGATGGTGATGGGCTTCCC-3′

### Rat I/R model

The I/R model was established in male SD rats as described previously [22]. Briefly, the rats were randomly divided into six groups: sham, I/R model, sham + pLKO.1, sham + pLKO.1-PLCE1, I/R + pLKO.1, I/R + pLKO.1-PLCE1, ten rats per group. Before I/R operation, the injection of pLKO.1 or pLKO.1-PLCE1 was performed as described previously [22]. The pLKO.1-PLCE1 or pLKO.1 was diluted with Entranster™ solution (Engreen Biosystem, Beijing, China) and 10% glucose mixture (1:1 v/v) to 0.5 μg/μl *in vivo*. Then, the rat was anesthetized and the thoracic cavity was exposed, a mixture was injected into the left ventricle apex and anterolateral wall at four different points (the similar points for other rats), 10 μl for each. The sham and I/R group rats were injected with an equal amount mixture of Entranster™ solution and 10% glucose. The rats were intramuscularly injected with 100000 units of penicillin for 4 consecutive days to prevent infection. Four days after injection, rats were subjected to myocardial I/R. Rats were anesthetized and ventilated with a rodent ventilator (Inspiras, MA, U.S.A.). The thoracic cavity was opened again carefully to expose the left anterior descending arteryata. Myocardial ischemia was induced by passing a 6-0 silk suture beneath the left anterior descending arteryata point 1–2 mm inferior to the left auricle. The suture was tightened for 45 min and then released for 180 min. The sham group only passed the suture but did not tighten. The suture was then tightened again, and the rats were intravenously injected with 2% Evans Blue. The hearts were immediately excised and stored at −20°C.

### Enzyme-linked immunosorbent assay

The heart tissues were cut into pieces and homogenized. The homogenates were centrifuged at 4°C at 10000×***g*** for 15 min and the supernatants were removed carefully. Cell culture supernatants were carefully collected at 24 h after H/R operation and centrifuged at 4°C at 10000×***g*** for 15 min. The cytokine (IL-1α, IL-6, TNF-α, and IL-10) concentrations of heart tissues supernatants or cell culture supernatants were detected by a commercial enzyme-linked immunosorbent assay (ELISA) kit according to the manufacturer’s instructions. The cytokine concentrations are expressed as picograms per milliliter.

### Immunohistochemistry

The heart tissues were fixed in 10% buffered paraformaldehyde for 24 h and embedded in paraffin. The paraffin-embedded tissues were cut into sections (4 μm). Then the heart sections were immersed in the target retrieval solution in water bath for 30 min. The endogenous peroxidase was blocked with 3% H_2_O_2_ for 15 min, and the nonspecific bindings were blocked with goat serum for 50 min. Then, the slides were stained with PLCE1 primary antibody and secondary antibody polymer HRP successively. Then the slices were stained with DAB and counterstained with Methyl Green. Images were taken under a microscope.

### Statistical analysis

All data were presented as means ± SD. Statistical analysis was conducted by one-way ANOVA with SPSS 13.0. Statistical significance was accepted at *P-*values <0.05.

## Results

### The expression of PLCE1 expression in H/R H9c2 cells and I/R rats

We established a model of cardiomyocytes injury *in vitro* by H/R in H9c2 cells. The effects of different duration of hypoxia time on H9c2 cells viability were detected by CCK-8 assay. As shown in Figure 1A, the cell viability decreased gradually with the hypoxia time increase, indicating the cardiomyocytes injury model was successful. Therefore, the mRNA and protein expression levels of PLCE1 were examined. As illustrated in Figure 1B, the mRNA and protein expression levels of PLCE1 in H9c2 cells were progressively increased along with the increase in H/R time. In addition, the expression of PLCE1 in another cardiomyocyte, HL-1 cells, under H/R condition was investigated. As shown in Figure 1C, the expression level of PLCE1 in H/R HL-1 cells was in accordance with results from H9c2 cells. To further confirm the expression of PLCE1 in myocardial I/R injury *in vivo*, a rat I/R model was established. As shown in Figure 1D, there was a low mRNA expression level of PLCE1 in the sham group, however, it was increased sharply in I/R group, approximately seven-fold compared with the sham group. Similarly, the protein expression level of PLCE1 in I/R group was also significantly higher than that in the sham group as determined by Western blot and IHC (Figure 1E,F). These results indicated that PLCE1 up-regulated in H/R H9c2 cells and I/R rats.

**Figure 1:** PLCE1 was up-regulated in H/R H9c2 cells and I/R rats (**A**) The H/R model in H9c2 cells was established by 2–24 h of hypoxia and 24 h of reoxygenation. The cell viability was detected by CCK-8 assay. (**B**) The expression level of PLCE1 in the H/R H9c2 cells was detected by qPCR and Western blot analysis. (**C**) The expression level of PLCE1 in the H/R HL-1 cells was detected by qPCR and Western blot analysis. (**D**) The mRNA expression level of PLCE1 in I/R rats was detected by qPCR analysis. (**E**) The protein expression level of PLCE1 in I/R rats was detected by Western blot analysis. (**F**) The expression of PLCE1 in I/R rats was detected by immunohistochemistry analysis. *P<0.05, **P<0.01, ***P<0.001 vs. Control group or Sham group.

### PLCE1 regulates inflammatory cytokines transcription and promotes NF-κB P65 phosphorylation

As previously reported, inflammation is involved in myocardial I/R injury, along with promoting the expression of pro-inflammatory cytokines [23,24]. So, the effect of overexpression or knockdown of PLCE1 on inflammatory cytokines (IL-6, TNF-α, IL-1α, and IL-10) in H/R H9c2 cells was investigated. A lentivirus vector carrying PLCE1 (pBabe-puro-PLCE1) was constructed and transfected into H9c2 cells prior to H/R to up-regulate the expression of PLCE1. The expression efficiency of PLCE1 as shown in Figure 2A,B. The mRNA and protein expression level of PLCE1 in pBabe-puro-PLCE1 group were increased more than 15-fold compared with that in the pBabe-puro group. Subsequently, we investigated the effect of pBabe-puro-PLCE1 on the expression of inflammatory cytokines IL-6, TNF-α, IL-1α, and IL-10 in H9c2 cells after H/R. As shown in Figure 2C, the expression and content of IL-6, TNF-α, and IL-1α were significantly increased and the anti-inflammatory cytokine IL-10 was decreased in H/R H9c2 cells compared with the control group. Overexpression of PLCE1 promoted the increase in IL-6, TNF-α, and IL-1α and the decrease in IL-10 significantly. In addition, the effect of knockdown of PLCE1 on inflammatory cytokines was also investigated. An shRNA against PLCE1 (pLKO.1-PLCE1) was used to interfere with the expression of PLCE1. As shown in Figure 2A,B, the relative expression levels of PLCE1 in the pLKO.1-PLCE1 group were reduced by more than 40% compared with that in the pLKO.1 group. As shown in Figure 2D, knockdown of PLCE1 decreased the expression of IL-6, TNF-α, and IL-1α and increased the IL-10 significantly.

**Figure 2:** PLCE1 regulates inflammatory cytokines expression and promotes NF-κB P65 phosphorylation (**A**) The mRNA expression level of PLCE1 after transfection with the pBabe-puro-PLCE1 or pLKO.1-PLCE1 in H9c2 cells. (**B**) The protein expression level of PLCE1 after transfected with pBabe-puro-PLCE1 or pLKO.1-PLCE1 in H/R H9c2 cells. (**C**) The expression and content of IL-6, TNF-α, IL-1α, and IL-10 after transfection with pBabe-puro-PLCE1 in H/R H9c2 cells were detected by qPCR and ELISA. (**D**) The expression and content of IL-6, TNF-α, IL-1α, and IL-10 after transfection with pLKO.1-PLCE1 in H/R H9c2 cells were detected by qPCR and ELISA. (**E**) The expression and phosphorylation of NF-κB P65 after transfected with pBabe-puro-PLCE1 or pLKO.1-PLCE1 in H/R H9c2 cells. (**F**) The expression and phosphorylation of NF-κB P65 in I/R rats. **P<0.01, ***P<0.001.

Studies have shown that activation of the NF-κB pathway plays an important role in the mediation of early inflammation during myocardial I/R injury [25,26]. Therefore, we evaluated the effect of PLCE1 on the activation of the NF-κB pathway. As shown in Figure 2E, there was no significant difference in the expression level of NF-κB P65 in each group. However, there was a significant change in NF-κB P65 phosphorylation. The increasing effect was also observed in I/R rats (Figure 2F). Overexpression of PLCE1 increased the NF-κB P65 phosphorylation while knockdown of PLCE1 decreased the NF-κB P65 phosphorylation.

### PLCE1 promotes NF-κB P65 phosphorylation via P38 and ERK1/2 pathways

In order to further elucidate the mechanism of PLCE1 on the regulation of NF-κB P65 phosphorylation, several key kinases which are probably involved in I/R injury, such as p38 and ERK1/2 from upstream MAPK signaling pathway were evaluated. As shown in Figure 3A,B, there was no significant difference in the protein expression levels of P38 and ERK1/2 in each group. However, phosphorylation of P38 (p-P38) and ERK1/2 (p-ERK1/2) was significantly increased after H/R, and further enhanced by overexpression of PLCE1. Knockdown of PLCE1 inhibited the phosphorylation of P38 and ERK1/2. Furthermore, an ERK1/2 inhibitor, PD98058, and a P38 inhibitor, SB203580, were used to verify the regulation effect of PLCE1 on NF-κB P65 signaling pathway. As shown in Figure 3C, the PD98058 decreased the phosphorylation of ERK1/2 that was enhanced by overexpression of PLCE1 but P38, while the SB203580 decreased the phosphorylation of P38 but ERK1/2. However, both of PD98058 and SB203580 decreased the phosphorylation of NF-κB P65. These results indicated that PLCE1 may activate NF-κB P65 signaling pathway via P38 and ERK1/2 phosphorylation.

**Figure 3:** PLCE1 promotes phosphorylation of P38 and ERK1/2 (**A**) The expression and phosphorylation of P38 and ERK1/2 after transfection with pBabe-puro-PLCE1 in H/R H9c2 cells. (**B**) The expression and phosphorylation of P38 and ERK1/2 after transfection with pLKO.1-PLCE1 in H/R H9c2 cells. (**C**) The effect of ERK1/2 inhibitor (PD98058) and P38 inhibitor (SB203580) on NF-κB P65 signaling pathway in H9c2 cells. **P<0.01, ***P<0.001.

### PLCE1 promotes the expression of inflammatory cytokines depending on the NF-κB signaling pathway

The previous data have proven that PLCE1 can promote the activation of NF-κB. So, a rescue experiment was used to determine whether PLCE1 promotes I/R injury is dependent on the NF-κB signaling pathway. A proven IKK inhibitor, IMD-0354, was used to suppress the NF-κB signaling pathway [27]. As shown in Figure 4A, overexpression of PLCE1 increased the phosphorylation of NF-κB P65, which was consistent with previous results. However, when IMD-0354 was added, the increase in NF-κB P65 phosphorylation caused by overexpression of PLCE1 was abrogated. Subsequently, the effect of IMD-0354 on the expression of inflammatory cytokines was also investigated. As shown in the Figure 4B, overexpression of PLCE1 significantly increased the expression of IL-6, TNF-α, and IL-1α and decreased the expression of IL-10. While, when NF-κB P65 phosphorylation was blocked by IMD-0354, the expressions of IL-6, TNF-α, and IL-1α were reduced and the expression of IL-10 was returned to be comparable with the control group (*P*>0.05).

**Figure 4:** PLCE1 promotes the expression of inflammatory cytokines depending on the NF-κB signaling pathway (**A**) IMD-0354 was used to suppress the NF-κB signaling pathway, and then the effect of pBabe-puro-PLCE1 on the expression and phosphorylation of NF-κB P65 in H/R H9c2 cells was determined. (**B**) The effect of pBabe-puro-PLCE1 and IMD-0354 on the expression and content of IL-6, TNF-α, IL-1α, and IL-10 in H/R H9c2 cells. ***P<0.001.

### Knockdown of PLCE1 attenuates inflammatory cytokine expression levels and inhibits NF-κB P65 phosphorylation in I/R rats

The I/R rat model was established to investigate the effects of PLCE1 on inflammation and NF-κB phosphorylation in I/R injury. An shRNA against PLCE1 was cloned into lentivirus vector pLKO.1 and injected into rats via intra-myocardial injection as previously reported [28]. As shown in Figure 5A, the expression of PLCE1 was increased significantly in I/R group compared with the sham group, and the expression of PLCE1 was knocked down efficiently by pLKO.1-PLCE1. In addition, the phosphorylation of NF-κB P65 was significantly increased in I/R group compared with the sham group. Knockdown of PLCE1 significantly inhibited NF-κB P65 phosphorylation. The inflammatory cytokines in I/R rat myocardial tissue were further determined. As shown in Figure 5B,C, the expression of IL-6, TNF-α, and IL-1α increased and the expression of IL-10 decreased sharply in I/R rat myocardial tissues compared with that of the sham group. Knockdown of PLCE1 significantly reduced the expression of IL-6, TNF-α, and IL-1α and increased the expression of IL-10. These results implied that PLCE1 regulates inflammation and NF-κB phosphorylation in I/R*.*

**Figure 5:** Effect of knockdown of PLCE1on inflammatory cytokine expression and NF-κB phosphorylation in I/R rats (**A**) The effect of pLKO.1-PLCE1 on the expression and phosphorylation of NF-κB P65 in I/R rats. (**B**-**C**) The effect of pLKO.1-PLCE1 on the expression and content of IL-6, TNF-α, IL-1α, and IL-10 in I/R rats. *P<0.05, **P<0.01, ***P<0.001.

## Discussion

The concept of myocardial I/R injury was first proposed by Hearse in 1977 [29]. Myocardial I/R injury refers to restore coronary flow on the basis of ischemic cardiac actually worsen or even lead to irreversible damage phenomenon. The clinical manifestations of myocardial I/R injury include reperfusion arrhythmia, myocardial infarction extension, cardiac insufficiency, and even sudden death after recanalization of the coronary arteries [30]. How to ensure the recovery of blood supply to ischemic myocardial tissue and avoiding or reducing myocardial I/R injury remains a critical problem in clinical practice. In the present study, an H/R-induced H9c2 cardiomyocytes injury and a rat model of myocardial I/R injury were used to evaluate the biological functions of PLCE1 and its underlying mechanism. First, we evaluated the expression level of PLCE1 in the H/R-induced H9c2 cells and I/R rats. Our results confirmed that the expression of PLCE1 was progressively increased along with the increase in hypoxia time in the H/R H9c2 cells. In the I/R rats, it presented a low expression of PLCE1 in the sham group, however, the expression PLCE1 was increased sharply in I/R group. These results indicated that PLCE1 up-regulated in H/R H9c2 cells and I/R rat myocardial tissue.

Myocardial I/R injury is a complex pathophysiological event involving multiple factors, it induces a strong acute inflammatory response which exacerbated after reperfusion, and recruits various inflammatory cells, monocytes, neutrophils and other cells to the ischemic area. These inflammatory cells secrete a variety of pro-inflammatory cytokines that ultimately promote myocardial damage [31]. Therefore, in order to elucidate the role of PLCE1 in myocardial I/R injury, we first examined the effect of PLCE1 on the inflammatory response. We constructed a PLCE1 overexpression lentivirus vector and an shRNA vector against PLCE1 to obtain different expression levels of PLCE1. The results showed that the PLCE1 was successfully up-regulated or down-regulated in H9c2 cells and I/R rats. Then the effects of different expression levels of PLCE1 on pro-inflammatory cytokines were examined. Our results suggested that up-regulation of PLCE1 promoted the expression of IL-6, TNF-α, and IL-1α and decreased the expression of IL-10, while knockdown of PLCE1 decreased the expression of IL-6, TNF-α, and IL-1α and increased the expression of IL-10. Similar results were also observed in I/R rats. These results indicated that PLCE1 is closely related to the inflammatory response in myocardial I/R injury.

Nuclear factor-κB (NF-κB) consists of a family of transcription factors that play critical roles in inflammation, immunity, cell proliferation, differentiation, and survival. The most common form of NF-κB is a heterodimer composed of P50 and P65 subunits [32]. Inducible NF-κB activation depends on phosphorylation-induced proteasomal degradation of the inhibitor of NF-κB proteins (IκBs), which retain inactive NF-κB dimers in the cytosol in unstimulated cells [32]. When suffering from myocardial I/R injury, the NF-κB was phosphorylated and released from the NF-κB/IκB complex after phosphorylation and degradation of IκB, the NF-κB translocates into the nucleus to initiate acute myocardial inflammation. Valen et al. found that NF-κB activity increased after 5 min of myocardial ischemia in a rat model [33]. Studies have shown that NF-κB plays a role in myocardial inflammation by promoting the expression of inflammatory factors and adhesion molecules [33]. In the present study, the effect of PLCE1 on the activation of the NF-κB pathway was evaluated. Our results showed that overexpression of PLCE1 increased the phosphorylation of NF-κB P65, while it was inhibited when the expression of PLCE1 was down-regulated. Similar results were observed in I/R rats. In addition, several key kinases, which may involve in NF-κB activation, such as P38 and ERK1/2 from the upstream MAPK signaling pathway were also evaluated. The results suggested that the overexpression of PLCE1 increased the phosphorylation of P38 and ERK1/2. In order to demonstrate whether PLCE1 promotes myocardial I/R injury is dependent on the NF-κB signaling pathway, a rescue experiment was conducted. The NF-κB signaling pathway was blocked by an IKK inhibitor, IMD-0354 [27]. The results showed that when IMD-0354 was added, the increase in NF-κB P65 phosphorylation induced by overexpression of PLCE1 was resisted. Furthermore, the regulation effect of overexpression of PLCE1 on the expression of cytokines (IL-6, TNF-α, IL-1α, and IL-10) was also antagonized by IMD-0354.

In conclusion, our study provided evidence that PLCE1 was up-regulated in H/R H9c2 cells and I/R rats. Overexpression of PLCE1 promoted the inflammatory via activation of the NF-κB signaling pathway.

## Abbreviations

AMI: acute myocardial infarction
CCK-8: Cell Counting Kit-8
DAG: diacylglycerol
H/R: hypoxia–reoxygenation
HRP: Horseradish Peroxidase
IFN: Interferongamma
IKK: IκB kinase
IL: Interleukin
IP3: inositol-1,4,5-triphosphate
IκB: inhibitor of NF-κB protein
I/R: ischemia–reperfusion
NF-κB: nuclear factor-κ B
PLCE1: phospholipase C ϵ-1
RIPA: Radio-immunoprecipation assay
SD: Standard deviation
